The article "Applicability of High-Frequency Ultrasound to the Early Diagnosis of Diabetic Peripheral Neuropathy" was retracted in 2024. Reasons: suspected computer-generated content; unreliable results or conclusions; concerns about the data; concerns about the results or conclusions.

# Applicability of High-Frequency Ultrasound to the Early Diagnosis of Diabetic Peripheral Neuropathy

**DOI:** 10.1155/2021/5529063

**Published:** 2021-03-18

**Authors:** Xishun Ma, Tongxia Li, Lizhen Du, Gang Liu, Ting Sun, Tongliang Han

**Affiliations:** ^1^Department of Ultrasound, Qingdao Municipal Hospital, Qingdao, Shandong 266071, China; ^2^Department of Tuberculosis, Qingdao Chest Hospital, Qingdao Central Medical Group, Qingdao, Shandong 266043, China

## Abstract

This study investigated the applicability of high-frequency ultrasound (HFU) to the early diagnosis of diabetic peripheral neuropathy (DPN). Patients with type 2 diabetes (*N* = 60) were divided into diabetic nonperipheral neuropathy and DPN groups (group A and group B, respectively; *n* = 30 each) based on electroneurophysiologic findings. Additionally, 30 nondiabetic patients were included as the healthy control group (group C). We calculated the cross-sectional area (CSA) of the median nerve (MN) of the right upper limb at 7 different sites (MN1–7) based on measured width (*W*) and thickness (*T*). Ultrasound imaging characteristics of the MN including internal echo, internal structure, boundary, epineurium, and blood flow were recorded. The 90 subjects (51 male and 39 female) had an average age of 56.09 ± 12.66 years. *W*, *T*, and CSA of the MN were increased in group A compared to group C (with significant differences at MN1, MN4, and MN7 (*P* < 0.05)) and in group B compared to group C (with significant differences at all 7 levels, especially MN6 and MN7 (*P* < 0.05)). Receiver operating characteristic curve analysis showed that CSA at the MN7 level had the highest diagnostic accuracy for DPN in group B, with a threshold value of 12.42 mm^2^. Ultrasound examination revealed that the MN had lost the internal sieve mesh structure and showed reduced echo, a partial blood flow signal, and thickened epineurium in patients with DPN; these findings were particularly obvious at MN6 and MN7, corresponding to the carpal tunnel. CSA was positively correlated with motor latency and F wave average latency and negatively correlated with motor conduction velocity, motor amplitude, and sensory conduction velocity in group B. Thus, HFU may be useful for the early diagnosis of DPN, which can improve clinical outcomes.

## 1. Introduction

Diabetic peripheral neuropathy (DPN) is one of the most common chronic complications of diabetes. At present, the diagnosis of DPN mainly depends on electroneurophysiologic examination, but this has drawbacks such as invasiveness and high costs in terms of time and resources. The development of high-frequency ultrasound (HFU) has permitted the analysis of the morphologic features of peripheral nerves, thus enabling early detection of lesions. In the present study, we examined the applicability of HFU to the early diagnosis of DPN by retrospective analysis of data from patients with DPN and diabetic nonperipheral neuropathy (DNPN).

The article "Applicability of High-Frequency Ultrasound to the Early Diagnosis of Diabetic Peripheral Neuropathy" was retracted in 2024. Reasons: suspected computer-generated content; unreliable results or conclusions; concerns about the data; concerns about the results or conclusions.

## 2. Materials and Methods

### 2.1. Participants

We analyzed data for 60 patients with type 2 diabetes who were admitted to the Endocrinology Department of Qingdao Municipal Hospital from October 2019 to October 2020 along with data for 30 healthy subjects collected during the same period. PASS software was used to calculate sample size. The ethics committee of the hospital approved the study, and informed consent was acquired from patients or families. The right upper limb median nerve was selected as the specific study object for the following reasons: no significant difference between unilateral and bilateral upper limbs and electrophysiological examination of the right upper limb. All patients met the 1999 World Health Organization diagnostic criteria for diabetes. Based on findings from the electroneurophysiologic examination, the patients were divided into DNPN and DPN groups (groups A and B, respectively); the 30 healthy subjects served as the control group (group C). Group A had 20 males and 10 females; group B had 19 males and 11 females; and group C had 12 males and 18 females. Patients with neuropathy caused by type 1 diabetes, lumbar spine disease, cerebrovascular disease, trauma, etc. were excluded. There were no statistically significant differences in age and sex ratios among the groups.

### 2.2. HFU Scan

The HFU linear array probe of a LOGIQ E8 (GE Healthcare, Little Chalfont, UK) or EPIQ 7 (Philips, Amsterdam, the Netherlands) ultrasound system was used for HFU scanning. The subject was in a supine position with right upper extremity abduction. The probe was placed vertically near the ulnar brachial artery of the subject's right upper limb to locate the median nerve (MN), which was measured at 7 different sites including 4–5 cm above the elbow (MN1), at the elbow joint (MN2), at the pronator teres entrance level (MN3), 4–5 cm above the transverse wrist stripes (MN4), at the transverse wrist stripes (MN5), at the pea bone level (MN6), and at the hook bone level (MN7). Vertical and cross-sectional scanning was performed. The width (*W*) and thickness (*T*) of the MN were measured and used to calculate the cross-sectional area (CSA). Additionally, changes in internal structure, echo, blood flow, and the epineurium at the 7 sites were recorded.

### 2.3. Electroneurophysiologic Examination

For neuroelectrophysiologic recordings, the patient was relaxed and in a supine position under constant temperature and quiet conditions. The following motor and sensory nerve conduction and F wave parameters were measured: distal motor latency (DML), mixed nerve action potential, motor conduction velocity (MCV), sensory nerve action potential, sensory conduction velocity (SCV), and F-wave average latency (F-AL).

The article "Applicability of High-Frequency Ultrasound to the Early Diagnosis of Diabetic Peripheral Neuropathy" was retracted in 2024. Reasons: suspected computer-generated content; unreliable results or conclusions; concerns about the data; concerns about the results or conclusions.

All operators were experienced doctors, and all measurements were obtained under double-blind test.

### 2.4. Statistical Analysis

Data are presented as mean ± standard deviation and were analyzed using SPSS v22.0 software (SPSS Inc., Chicago, IL, USA). Single-factor analysis of variance and the *t*-test were used to compare quantitative data, and the chi-squared test was used for categorical variables. Receiver operating characteristic (ROC) curve analysis was carried out to determine the optimal threshold value for accurate diagnosis of DPN. Correlation analysis was performed by linear regression. Differences with *P* < 0.05 were considered statistically significant.

## 3. Results

### 3.1. Comparison of MN Ultrasound Measurements between Groups

The size of the MN in group C decreased from the proximal part to the distal end. *W*, *T*, and CSA of the MN were increased in group A compared to group C, with significant differences at MN1, MN4, and MN7 (*P* < 0.05). Similarly, *W*, *T*, and CSA of the MN were increased in group B compared to groups C and A, with significant differences at all 7 levels but especially at MN6 and MN7 (*P* < 0.05) (Tables 1 and 2).

### 3.2. ROC Curve Analysis of CSA at Different Sites along the MN in DPN Patients

Patients with DPN had larger area under the ROC curve (AUC) for CSA of the MN than the other groups, with higher specificity and sensitivity at MN6 and MN7 than at other levels. MN6 and MN7 corresponded to the carpal tunnel. MN7 had the highest AUC at 0.88, with a sensitivity and specificity of 0.73 and 0.88, respectively; thus, the diagnostic accuracy was the highest at the MN7 level. The optimal threshold value of CSA was 12.42 mm^2^ (Figure 1 and Table 3).

### 3.3. HFU Features of the MN

The results of HFU scans showed that the MN in group C had a mesh-like structure in cross section, with a clear internal structure and boundary, uniform thickness of the epineurium, and parallel bands of high and low echoes in vertical sections (Figure 2). There was no obvious blood flow in the nerve. Compared to group C, in groups A and B, the internal sieve mesh structure of the MN was lost (group A, 76.7%; group B, 96.7%; and group C, 36.7%); moreover, the echo was reduced (group A, 66.7%; group B, 96.7%; group C, 36.7%) and there was a partial blood flow signal (group A, 26.7%; group B, 40%; and group C, 6.7%), accompanied by a thickened epineurium. These HFU findings were especially obvious at MN6 and MN7 (hook bone level). The MN in groups A and B showed significant reductions in the internal sieve mesh structure, echo, and blood flow compared to group C (*P* < 0.05); and between groups A and B, the differences in the decreased internal echo and loss of mesh structure were significant (*P* < 0.05), whereas blood flow signals were comparable (*P* > 0.05) (Table 4).

The article "Applicability of High-Frequency Ultrasound to the Early Diagnosis of Diabetic Peripheral Neuropathy" was retracted in 2024. Reasons: suspected computer-generated content; unreliable results or conclusions; concerns about the data; concerns about the results or conclusions.

### 3.4. Correlation Analysis between HFU Measurements and Electroneurophysiologic Parameters in DPN Patients

The CSA of the MN in the DPN group was positively correlated with DML and F-AL and negatively correlated with MNAP, MCV, and SCV (Table 5).

## 4. Discussion

DPN is one of the most common chronic complications of diabetes, developing in more than half of patients [1]. The main clinical manifestations are symmetric pain, numbness, loss or disappearance of pain and temperature sensitivity, muscle weakness, and muscle atrophy of bilateral extremities as well as typical glove- and sock-like sensory disorders [2, 3]. DPN has an insidious onset and high incidence, and its pathologic severity is not proportional to clinical symptoms, as many patients are asymptomatic for a long time. It has been reported that 10% of newly diagnosed type 2 diabetes patients already have peripheral neuropathy when the disease course is >10 years [4], and more than 50% of patients develop varying degrees of DPN, which is associated with serious complications such as foot gangrene and ulcers that can seriously affect the quality of life of patients. Therefore, early diagnosis of DPN is critical to ensure a good clinical outcome.

The pathogenesis of DPN is unclear; because of the existence of many types of peripheral neuropathy, it is difficult to explain all of the pathologic features by a single mechanism. Long-term hyperglycemia metabolic disorder and microvascular disease are the major risk factors; others include changes in nerve growth factor level, peroxide- and free radical-induced damage, and abnormal metabolism of essential fatty acids [5].

At present, the diagnosis of DPN mainly relies on clinical manifestations and electroneurophysiologic findings. However, by the time the patient shows clinical symptoms, there are already obvious lesions in the peripheral nerves and early intervention is not possible. Electroneurophysiologic examination is the gold standard for DPN diagnosis, but it is time-consuming, laborious, costly, and invasive and is thus unsuitable for routine DPN screening [6]. With advances in ultrasound technology in recent years including probes with higher frequency and better resolution, it has become possible to visualize internal structures such as the epineurium, perineurium, and nerve bundles with a diameter of ≤0.5 mm as well as some small nerves and cutaneous nerves. Thus, HFU provides valuable morphologic information that can complement electrophysiologic data [7, 8].

The article "Applicability of High-Frequency Ultrasound to the Early Diagnosis of Diabetic Peripheral Neuropathy" was retracted in 2024. Reasons: suspected computer-generated content; unreliable results or conclusions; concerns about the data; concerns about the results or conclusions.

In this study, we compared the features of the MN of the right upper limb in patients with DPN or DNPN and healthy control subjects, including changes in size, internal echo, structure, and blood flow. In healthy subjects, CSA and anteroposterior diameter of the MN were reduced compared to the elbow joint, especially at the level of the carpal tunnel; and the shape was also changed from round or oval to flat oval. The *W*, *T*, and CSA at the 7 measured sites along the MN were increased in DNPN and DPN patients compared to controls; the differences were statistically significant. The level of aldose reductase was shown to be elevated in DPN, resulting in excessive conversion of glucose to sorbitol and fructose accumulation [9]. Sorbitol and fructose are hypertonic molecules that can increase osmotic pressure in nerve cells and cause water and sodium retention and nerve swelling and thickening, which are all pathophysiologic effects.

Comparing group B with group A, the differences were only statistically significant at the level of the carpal tunnel (MN6, MN7). In our ROC curve analysis, the AUC was largest at the level of MN7 (hook bone), and the optimal threshold value for CSA was 12.42 mm^2^. The MN exits the carpal tunnel at the level of the hook bone. The carpal tunnel contains abundant flexor tendons that can easily compress the nerve. When the MN is lesioned and degenerates in patients with DPN, it can be vulnerable to compression and edematous or thickened. Additionally, in patients with DPN, the internal sieve-like structure of the MN was lost and echo was reduced by HFU. The pathologic basis for these effects may be the hyperglycemic state of DPN patients, which resulted in a decreased blood supply to the nerve and hypoxia. The blood supply and nutrition of nerve fiber bundles depend on the tunica intima, which was the most affected structure. When complicated with peripheral neuropathy, hyperglycemia can cause nerve cells to swell, disintegrate, and demyelinate [10].

The ultrasound findings were more prominent at the level of the carpal tunnel because under normal circumstances, this area is affected by the carpal bone; thus, the probe was unable to remain in a vertical position relative to the cut nerve surface at all times, causing the echo of the MN to be lower at the carpal tunnel than at the upper arm. Moreover, the internal mesh-like structure was less clear in the former than in the latter, which was further aggravated under pathologic conditions. We also found that the peripheral and internal blood flow rates of the MN were relatively low. Blood flow in the MN was observed in 40% of DPN patients, which was higher than the rate in the other two groups. This may be attributable to the fact that blood flow in the endoneurium and perineurium is increased due to the enhancement of vascular reactivity in the early stage of diabetes but is decreased as a result of vascular sclerosis in the late stage [11].

The article "Applicability of High-Frequency Ultrasound to the Early Diagnosis of Diabetic Peripheral Neuropathy" was retracted in 2024. Reasons: suspected computer-generated content; unreliable results or conclusions; concerns about the data; concerns about the results or conclusions.

The CSA of the MN showed positive and negative correlations with electroneurophysiologic parameters in patients with DPN, indicating that HFU can to some extent reveal changes in the functional properties of nerves. Moreover, it can clearly display the anatomic position of nerves and their relationship to adjacent structures as well as morphologic changes. Thus, HFU can aid in the early diagnosis of DPN by allowing lesions to be detected at an early stage, which can improve clinical outcomes.

Because the gold standard for diagnosing DPN is neurophysiological examination, our diagnosis of DPN may be not accurate enough because of small samples. Therefore, large simples are needed for further confirmation.

## Figures and Tables

**Figure 1:** ROC curve for CSA of the MN at MN7 in DPN patients.

**Figure 2:** Representative HFU images of the MN. (a, b) In group C, the MN showed a sieve mesh structure in cross section (a) and parallel bands of high and low echoes (b). (c, d) In a 68-year-old male patient in group B, the sieve mesh structure of the MN was lost and the internal echo was decreased at the level of MN6 in cross section (c); the MN showed increased blood flow at MN6 and MN7 in vertical sections (d). (e, f) In a 60-year-old male patient in group B, the MN had a thickened epineurium at the level of MN7 in cross section (e) and there was no blood flow in vertical sections (f).

**Table 1:** *W*, *T*, and CSA of the median nerve at different levels in the 3groups.

MN level	Group A			Group B			Group C		
	*W*	*T*	CSA	*W*	*T*	CSA	*W*	*T*	CSA
MN1	4.91 ± 0.70	2.93 ± 0.39	11.31 ± 2.33	5.00 ± 0.46	3.09 ± 0.51	12.19 ± 2.52	4.51 ± 0.49	2.80 ± 0.33	9.88 ± 1.33
MN2	4.91 ± 0.65	2.71 ± 0.35	10.49 ± 1.98	5.26 ± 0.68	2.92 ± 0.48	11.99 ± 2.42	4.60 ± 0.57	2.68 ± 0.39	9.66 ± 1.72
MN3	4.42 ± 0.69	2.23 ± 0.39	7.75 ± 1.92	4.81 ± 0.68	2.29 ± 0.44	8.66 ± 2.05	4.30 ± 0.65	2.08 ± 0.32	7.05 ± 1.63
MN4	4.20 ± 0.57	2.61 ± 0.52	8.61 ± 2.03	4.38 ± 0.69	2.65 ± 0.37	9.11 ± 1.91	3.90 ± 0.54	2.40 ± 0.34	7.36 ± 1.59
MN5	5.96 ± 1.02	2.21 ± 0.30	10.36 ± 2.33	6.44 ± 0.70	2.35 ± 0.31	11.91 ± 2.20	5.70 ± 0.64	2.11 ± 0.25	9.45 ± 1.76
MN6	5.68 ± 0.75	2.33 ± 0.23	10.37 ± 1.64	6.64 ± 0.66	2.50 ± 0.30	13.09 ± 2.04	5.79 ± 0.72	2.11 ± 0.30	9.62 ± 1.96
MN7	6.01 ± 0.76	2.47 ± 0.28	11.48 ± 1.71	6.77 ± 0.60	2.55 ± 0.25	13.57 ± 1.71	5.44 ± 0.90	2.08 ± 0.42	8.87 ± 2.28

CSA: cross-sectional area (mm^2^); MN: median nerve; *T*: thickness (mm); *W*: width (mm).

The article "Applicability of High-Frequency Ultrasound to the Early Diagnosis of Diabetic Peripheral Neuropathy" was retracted in 2024. Reasons: suspected computer-generated content; unreliable results or conclusions; concerns about the data; concerns about the results or conclusions.

**Table 2:** Comparisons of *W*, *T*, and CSA at different levels of the median nerve between groups (*t*-test).

MN level	*W*		*T*		CSA	
	*t* statistic	*P*	*t* statistic	*P*	*t* statistic	*P*
Group A vs. group C						

MN1	2.53	0.010	1.41	0.170	2.93	≤0.001
MN2	1.99	0.050	0.32	0.750	1.73	0.080
MN3	0.71	0.480	1.58	0.120	1.53	0.130
MN4	2.13	0.030	1.84	0.070	2.65	0.010
MN5	1.19	0.230	1.41	0.160	1.72	0.090
MN6	−0.57	0.570	3.17	≤0.001	1.60	0.110
MN7	2.65	0.010	4.14	≤0.001	5.01	≤0.001

Group B vs. group C						

MN1	3.95	≤0.001	2.66	0.010	4.43	≤0.001
MN2	4.07	≤0.001	2.11	0.040	4.29	≤0.001
MN3	2.98	≤0.001	2.08	0.040	3.38	≤0.001
MN4	2.97	≤0.001	2.78	≤0.001	3.84	≤0.001
MN5	4.29	≤0.001	3.39	≤0.001	4.79	≤0.001
MN6	4.75	≤0.001	5.04	≤0.001	6.71	≤0.001
MN7	6.80	≤0.001	5.21	≤0.001	9.05	≤0.001

Group A vs. group B						

MN1	0.60	0.550	1.39	0.170	1.40	0.170
MN2	2.03	0.040	1.91	0.060	2.62	0.010
MN3	2.22	0.030	0.58	0.570	1.77	0.080
MN4	1.06	0.290	0.42	0.680	0.97	0.330
MN5	2.13	0.030	1.83	0.070	2.64	0.010
MN6	5.23	≤0.001	2.46	0.020	5.68	≤0.001
MN7	4.33	≤0.001	1.17	0.250	4.75	≤0.001

CSA: cross-sectional area (mm^2^); MN: median nerve; *T*: thickness (mm); *W*: width (mm).

**Table 3:** Receiver operating characteristic curve analysis for the cross-sectional area at different levels of the median nerve in diabetic peripheral neuropathy patients.

MN level	AUC	Sensitivity	Specificity	Optimal threshold for CSA
MN1	0.69	0.53	0.80	12.05
MN2	0.72	0.50	0.82	11.79
MN3	0.70	0.67	0.67	7.85
MN4	0.67	0.77	0.57	7.62
MN5	0.75	0.90	0.57	9.86
MN6	0.87	0.93	0.70	10.71
MN7	0.88	0.73	0.88	12.42

AUC, area under the receiver operating characteristic curve; CSA: cross-sectional area (mm^2^); MN: median nerve; *T*: thickness (mm); *W*: width (mm).

**Table 4:** Analysis of ultrasonographic features at the MN7 level of the median nerve.

	Blood flow		Mesh structure		Internal echo	
	With	Without	With	Without	Reduction	No change
Group C vs. group A						

Group C	2	28	19	11	11	19
Group A	8	22	7	23	20	10
*χ* ^2^	4.32		9.77		5.41	
*P*	0.040		≤0.001		0.020	

Group C vs. group B						

Group C	2	28	19	11	11	19
Group B	12	18	1	29	29	1
*χ* ^2^	9.32		24.30		24.30	
*P*	≤0.001		≤0.001		0.010	

Group B vs. group A						

Group A	8	22	7	23	20	10
Group B	12	18	1	29	29	1
*χ* ^2^	1.20		5.19		9.02	
*P*	0.210		0.030		≤0.001	

**Table 5:** Correlation analysis between the cross-sectional area of the median nerve and neurophysiologic parameters at MN7 in diabetic peripheral neuropathy patients.

	DML	MNAP	MCV	F-AL	SNAP	SCV
*R*	0.61	−0.78	−0.56	0.51	−0.17	−0.54
*P*	≤0.001	≤0.001	≤0.001	≤0.001	0.380	≤0.001

DML: distal motor latency; F-AL: F-wave average latency; MCV: motion conduction velocity; MNAP: mixed nerve action potential; SCV: sensory conduction velocity; SNAP: sensory nerve action potential.

The article "Applicability of High-Frequency Ultrasound to the Early Diagnosis of Diabetic Peripheral Neuropathy" was retracted in 2024. Reasons: suspected computer-generated content; unreliable results or conclusions; concerns about the data; concerns about the results or conclusions.

## Data Availability

All data generated or used in this study can be found in the article.
